The article "Injuries and outcomes resulting due to falls in elderly patients presenting to the Emergency Department of a tertiary care hospital – a cohort study" was retracted in 2023. Reasons: errors in the text; plagiarized data; lack of ethics approval or compliance; no approval from a third party.

# Injuries and outcomes resulting due to falls in elderly patients presenting to the Emergency Department of a tertiary care hospital – a cohort study

**DOI:** 10.1186/s12873-023-00784-z

**Published:** 2023-02-10

**Authors:** Salman Muhammad Soomar, Zeyanna Dhalla

**Affiliations:** 1 Department of Emergency Medicine, Aga Khan University, Karachi, Pakistan; 2 University of Michigan, Ann Arbor, Michigan, USA

**Keywords:** Fall, Elderly, Injuries, Emergency

## Abstract

**Background:**

Fall injuries and trauma-related hospitalizations are the most common causes of injury and in-hospital stay amongst the elderly population. After the age of 65, the severity and frequency of fall-related problems increases; the repercussions are challenging for senior citizens, caregivers, and healthcare professionals. This study aims to determine the injuries and outcomes resulting from falls in elderly patients presenting to Emergency Department of a tertiary care hospital.

**Methods:**

A cohort study design was used. All elderly patients aged ≥ 60 years who visit the Emergency Department with a history of a fall as a primary complaint presenting to the ED of a tertiary care hospital in Karachi, Pakistan were included. A purposive sampling strategy was used to enroll 318 patients from August 2021 to February 2022. The outcome was risk of mortality. Each individual was followed for 90 days to study the outcome. A multivariable logistic regression was applied to check the association between the outcome and covariates. Crude and adjusted risk ratios were reported. A *p*-value ≤ 0.05 was considered significant.

**Results:**

Of the 318 participants, 265 (83.3%) were fall injury patients with comorbidities. More than half of the patients in both groups were female [32 (60.4%) & 146 (55.1%)]. Eyeglasses were used by most of the fall patients both without and with comorbidities [21 (39.6%) & 152 (57.4%) *p* 0.018]. There were multiple reasons for a fall including imbalance/dizziness, which was reported by one third of participants in both groups [15 (28.3%) & 77 (29.1%)] followed by a fall from stairs/steps/escalator [15 (28.3%) & 44 (16.6%) *p* 0.005]. At the end of one month, of those who had a comorbidity 20 (7.5%) expired. The risk of mortality among fall related injuries in elderly patients who were more than 80 years was 1.48 times (95% CI: 1.20–2.10) more likely when compared to those patients who were younger than 80 years.

**Conclusion:**

Efforts should be made to improve management of the underlying etiology of falls to prevent them in future. The factors that contribute to falls should be identified. Strategies and interventions should be planned to mitigate this risk of fall in elderly to improve their quality of life.

The article "Injuries and outcomes resulting due to falls in elderly patients presenting to the Emergency Department of a tertiary care hospital – a cohort study" was retracted in 2023. Reasons: errors in the text; plagiarized data; lack of ethics approval or compliance; no approval from a third party.

## Introduction

The elderly population faces an increased burden of fall related injury and mortality. This creates a major public health concern and burdens this population with a risk of longstanding pain, disability, functional impairments, and death [1]. There is a worldwide increase in the elderly population and falls are a major global health problem in this age group. According to Centre for Disease Control (CDC), falls are the leading cause of injury-related death among adults aged 65 years and older [2]. It has been noted that injuries related to falls, in the elderly population, are the leading cause of disabilities and death. The World Health Organization (WHO) has estimated a total of 424,000 falls per year, globally, and around 37.3 million falls have required medical attention. The elderly population accounts for 12% to 24% of all visits to ED [1, 3]. When compared to younger populations, the elderly have much higher rates of mortality after a low impact fall. Not only are there higher levels of mortality among this demographic, but these patients also have higher rates of hospitalizations and longer hospital stays than younger demographics [4]. Falls are estimated to be the thirteenth leading cause of worldwide deaths in 2015. The global burden of disease report has estimated that fall-related deaths have increased by 55%—from 348,000 deaths annually in 1990 to about 540,000 deaths in 2015 [5]. The point of concern is that the burden is disproportionately distributed as more than 82% of fall-related mortality and 92% of disability adjusted life year (DALY) loss occurred in low- and middle-income countries. WHO attributed over 80% fall-related fatalities occurred in low- and middle- income countries. It is a matter of concern for emergency settings because emergency departments (EDs) are the first and most common point of health care access for elderly people [6]. In 2019 alone, 3 million elderly patients visited the ED due to a fall related injury. This issue is only going to grow in the coming years, as life expectancy is increasing, thus there will be higher numbers of individuals over the age of 65 across the globe [4].

The studies conducted in the United Kingdom (UK), Canada and United States (US) reported the prevalence of falls in the elderly to be around 30%, 20%, and 12% respectively [7]. In United States, the overall rate of older adult deaths from falls increased from 31% in 2007 to 40% in 2016 (3.0% per year) [8]. Various European countries showed that the number of deaths is significantly increasing up to 20% per year [9]. Roche et al. found the mortality risk after a fall is 9.6% during the first 30 days and 33% after a period of one year. The one-year cumulative mortality for individuals hospitalized due to a fall causing fracture was 25.2% (63 deaths) [10]. In regional studies, non-fatal injuries were more prevalent than fatal. A study conducted in India also showed that mortality after a fall is 25% [11]. In 2016, a study conducted at an Emergency Department in Turkey demonstrated a prevalence rate of 45% (*n* = 148) [12]. The age standardized mortality of elderly falls in a study done in mainland China from 2013 to 2020 has shown an increase in falls over the years [13]. A national study at Karachi, Pakistan reported 45% (*n* = 100) of falls among the elderly had significant associated factors such as a previous history of fall, activity of daily living, comorbidities and medications [14]. A study conducted in the Emergency Department of Rawalpindi, Pakistan stated the prevalence of falls to be 45% out of which mortality was reported at 17% in males and 12.9% in females.

The article "Injuries and outcomes resulting due to falls in elderly patients presenting to the Emergency Department of a tertiary care hospital – a cohort study" was retracted in 2023. Reasons: errors in the text; plagiarized data; lack of ethics approval or compliance; no approval from a third party.

There is a scarcity of local data on injuries and mortality related to falls among elderly visiting the Emergency Department. Falls in the elderly population is a major public health problem because it leads to premature mortality and those who survive sustain significant losses to their quality of life. Effective public health interventions have been found to reduce this incidence of falls and prevent further complications. Unfortunately, there is paucity of data on injury and mortality trends after a fall in the elderly from this region. We propose to fill this gap by conducting a study that aims to determine the injuries and outcomes resulted due to fall in elderly patients presenting to the Emergency Department of a tertiary care hospital.

### Operational definitions

#### Fall

A fall is defined as an event which results in a person coming to rest inadvertently on the ground or floor or other lower level [15].

### Fall related injury

An injury related to a fall includes fracture, laceration, contusion, chipped tooth, soft tissue injury, pain, head or brain injury, or death [16].

## Methods

### Study design

This was a cohort study. Exposure was considered history of fall or fall-related injuries as a primary complaint. The outcome was risk of mortality. All these individuals were followed for 90 days to the study outcome.

### Study setting

This study was conducted at the ED of the Aga Khan University Hospital, Karachi Pakistan (AKUH). It is a tertiary care hospital in Karachi and caters a vast population of Pakistan and Afghanistan with different socio-economic statuses. The ED has an occupancy of 60 patients.

### Study population

All elderly patients aged ≥ 60 years who visited the Emergency Department with a history of a fall as a primary complaint.

The article "Injuries and outcomes resulting due to falls in elderly patients presenting to the Emergency Department of a tertiary care hospital – a cohort study" was retracted in 2023. Reasons: errors in the text; plagiarized data; lack of ethics approval or compliance; no approval from a third party.

### Eligibility criteria

All elderly individuals aged ≥ 60 years with a history of a fall as a presenting complaint or reason to visit the Emergency Department and provided informed written consent by the caregiver or family.

### Sampling technique and sample size

A purposive sampling strategy was used to enroll the patients. The sample size was calculated using the 95% Confidence Interval (CI) and 80% power with a 1:2 exposed to unexposed ratio. The risk of mortality among elderly with fall was 17% according to Bhatti, Junaid A., et al. 2015. The sample size calculated was 289. After adjusting 10% for non –respondent rate, the final sample size was 318.

### Data collection and management

The data was collected by trained data collectors. Informed written consent was obtained from caregivers or family members. Patients or their caregivers were asked to answer a questionnaire related to possible factors that possibly caused the fall related injury. Pilot testing was done on 25 patients. The content validity of the tool was calculated as 0.72 after the review of 4 experts. The reliability of the tool was 0.88 which was obtained through Cronbach alpha. All patients aged ≥ 60 years with a history of falls who presented to the ED from August 4, 2021 to Feb 28, 2022 have been included. Data was collected on socio-demographic factors, lifestyle/behavioral factors, addictions/habits/substance use/misuse, functional classification, previous history of fall, comorbidities, and medication history. The outcome was risk of mortality. All these individuals were followed for 90 days. The first follow up was done at 30 days and final at 90 days. Patients were contacted by the telephone for mortality, revisits, and functional status.

Data was collected and entered in the Redcap software; double data entry was done to rectify errors. Missing information was rechecked and asked for from patients’ caregivers.

### Statistical analysis

Data was analyzed using Stata version 16. Descriptive analysis i.e., frequencies and percentages were calculated for categorical variables such as age, gender, family history, education, socioeconomic status, medical comorbidities (hypertension, diabetes mellitus, stroke etc.). Data was stratified on comorbidities. Post stratification Chi-square test were applied to check the association between qualitative categorical independent variables and comorbidities. Fisher’s exact test was applied for the non-parametric data where frequencies were ≤ 5. The outcome variable was binary; therefore, the multivariable logistic regression was applied to check the association between outcome and covariates. Crude and adjusted risk ratio were reported. A *p* value ≤ 0.05 was considered significant.

The article "Injuries and outcomes resulting due to falls in elderly patients presenting to the Emergency Department of a tertiary care hospital – a cohort study" was retracted in 2023. Reasons: errors in the text; plagiarized data; lack of ethics approval or compliance; no approval from a third party.

## Results

Of the *n* = 318 participants, most of the patients with injuries secondary to fall were with comorbidities *n* = 265 (83.3%) whereas *n* = 53 (16.7%) was without comorbidities. More than half of the patients in both the groups were females [*n* = 32 (60.4%) & 146 (55.1%)]. Most of the patients were from the old age group, with a majority lying between 65–80 years [24 (45.3%) to 143 (54.0%)] respectively. More than 85% of the patients were unemployed in both fall without and with comorbid group [46 (86.8) & 232 (87.5)]. One third of the patients in these groups were graduates [18 (34.0%) & 99 (37.4)]. Most of the patients with comorbidities were taking anti-HTN 2b medicine 62 (23.4%) followed by anti-diabetic medicine 61 (23.0%) Almost all of the included patients with or without comorbidities were able to perform daily activities. Similarly, they were also able to perform instrumental activities of daily life such as shopping, housekeeping, and keeping their accounts in order. In assisting aids, the majority wore eyeglasses either without or with comorbidities [21 (39.6%) & 152 (57.4%) *p* 0.018]. Memory assessment was done for 173 (54.4%) of the total patients out of which 30 (56.6%) were without comorbid and 117 (81.8%) were with comorbid, had a score of ≥ 3 (see Table 1).

**Table 1:** Baseline characteristics of elderly patients with fall related injuries and risk of mortality (*n* = 318)

Characteristics	Total	Comorbidities *n* (%)		*p*-value
		**Fall** **(Without Comorbidity)**	**Fall** **(With Comorbidity)**	
	**318**	**53 (16.7%)**	**265 (83.3%)**	
**Gender**				
Male	140 (44)	21 (39.6)	119 (44.9)	0.479
Female	178 (56)	32 (60.4)	146 (55.1)	
**Age (years)**				
< = 65 Years	84 (26.4)	18 (34)	66 (24.9)	0.366
66–80 Years	167 (52.5)	24 (45.3)	143 (54.0)	
> 80 Years	67 (21.1)	11 (20.8)	56 (21.1)	
**Employment Status**				
Unemployed	278 (87.4)	46 (86.8)	232 (87.5)	0.212
Employed	32 (10.1)	5 (9.4)	27 (10.2)	
Own shop Rent	1 (0.3)	1 (1.91)	0 (0)	
Housewife	3 (0.9)	0 (0)	3 (1.1)	
Retired	4 (1.3)	1 (1.9)	3 (1.1)	
**Education**				
Illiterate	56 (17.6)	10 (18.9)	46 (17.4)	0.967
Primary	54 (17)	8 (15.1)	46 (17.4)	
Secondary	61 (19.2)	11 (20.8)	50 (18.9)	
Intermediate	29 (9.1)	6 (11.3)	23 (8.7)	
Graduation	117 (36.8)	18 (34.0)	99 (37.4)	
Madrasa	1 (0.3)	0 (0)	1 (0.4)	
**History of medication**				
Anti-diabetic	61 (23.0)	-	61 (23.0)	-
Anti HTN 2a	15 (5.7)	-	15 (5.7)	
Anti HTN 2b	62 (23.4)	-	62 (23.4)	
Diuresis 2c	6 (2.3)	-	6 (2.3)	
Anti-bedrest	16 (6.0)	-	16 (6.0)	
Other	54 (20.4)	-	54 (20.4)	
**Activity of Daily Living**				
Eating	304 (95.6)	51 (96.2)	253 (95.5)	0.226
Changing	300 (94.3)	51 (96.2)	249 (94)	
Bath	296 (93.1)	51 (96.2)	245 (92.5)	
Walk	294 (92.5)	51 (96.2)	243 (91.7)	
Using toilet	293 (92.1)	51 (96.2)	242 (91.3)	
**Instrumental Activity of Daily Living**				
Shopping	221 (69.5)	43 (81.1)	178 (67.2)	0.307
Housekeeping	213 (67.0)	43 (81.1)	170 (64.2)	
Accounts	213 (67.0)	44 (83)	169 (63.8)	
Preparing Food	198 (62.3)	42 (79.2)	156 (58.9)	
Transportation	200 (62.9)	42 (79.2)	158 (59.6)	
**Assisting Aid**				
Eyeglasses	173 (54.4)	21 (39.6)	152 (57.4)	0.018*
Walking aids	82 (25.8)	7 (13.2)	75 (28.3)	
Hearing aids	41 (12.9)	5 (9.4)	36 (13.6)	
**Memory assessment**				
Yes	173 (54.4)	30 (56.6)	143 (54)	< 0.001*
**Scoring Criteria**				
≥ 3	147 (85.0)	30 (56.6)	117 (81.8)	0.011*
< 3	26 (15.0)	0 (0)	26 (18.2)	

^*^Significant

A previous history of falls was reported to be *n* = 8 (15.1%) in patients who had no comorbid, and *n* = 84 (31.7%) in patients with comorbid (*p* 0.015). Most of the patients reported their fall to occur at home in both groups [*n* = 18 (34.0%) & *n* = 144 (54.7) *p* 0.001] and the floor type was commonly observed to be tiles [*n* = 218 (68.6%) & *n* = 184 (69.4)]. There were multiple reasons for the fall such as disbalance/dizziness which was reported by one third of the participants in both the groups [*n* = 15 (28.3%) & *n* = 77 (29.1%)] followed by fall from stairs/steps/escalator [*n* = 15 (28.3%) & *n* = 44 (16.6%) *p* 0.005]. Most of the falls occurred in the morning in patients with comorbid *n* = 167 (63.0%) while most of the falls happened in the evening time in falls without comorbid group *n* = 44 (83.0%). Upper extremities [15 (29.4%) & 46 (18.5%)] and lower extremities [19 (37.3) & 77 (31.0)] were majorly injured due to fall in both the groups (see Table 2).

The article "Injuries and outcomes resulting due to falls in elderly patients presenting to the Emergency Department of a tertiary care hospital – a cohort study" was retracted in 2023. Reasons: errors in the text; plagiarized data; lack of ethics approval or compliance; no approval from a third party.

**Table 2:** Fall related characteristics of elderly patients with fall related injuries and risk of mortality (*n* = 318)

Characteristics	Total	Comorbidities *n* (%)		*p*-value
		**Fall** **(Without Comorbidity)**	**Fall** **(With Comorbidity)**	
	**318**	**53 (16.7%)**	**265 (83.3%)**	
**Previous fall**				
Yes	92 (28.9)	8 (15.1)	84 (31.7)	0.015*
**Living Alone**				
Yes	11 (3.5)	1 (1.9)	10 (3.8)	0.493
**Place of fall**				
Home	163 (51.3)	18 (34.0)	144 (54.7)	0.001*
Bathroom	72 (22.6)	12 (22.6)	60 (22.6)	
Stairs	21 (6.6)	6 (11.3)	15 (5.7)	
Road /outside home	26 (8.2)	6 (11.3)	20 (7.5)	
Parking area	4 (1.3)	0 (0)	4 (1.5)	
Prayer Place	8 (2.5)	3 (5.7)	5 (1.9)	
Ground	10 (3.1)	3 (5.7)	7 (2.6)	
Hospital	5 (1.6)	0 (0)	5 (1.9)	
Other	9 (2.8)	5 (9.4)	4 (1.5)	
**Floor type**				
Tile	218 (68.6)	34 (64.2)	184 (69.4)	0.025*
Concrete	52 (16.4)	11 (20.8)	41 (15.5)	
Carpets	18 (5.7)	3 (5.7)	15 (5.7)	
Cement	6 (1.9)	0 (0)	5 (1.9)	
Other	27 (8.55)	5 (9.4)	22 (8.3)	
**Reason of fall**				
Disbalance/Dizzy	92 (28.9)	15 (28.3)	77 (29.1)	0.005*
Stroke/ Seizures	3 (0.9)	0 (0)	3 (1.1)	
Weakness	46 (14.5)	3 (5.7)	43 (16.2)	
Visual (Blinded)	9 (2.8)	3 (5.7)	6 (2.3)	
Rough surface	32 (10.1)	11 (20.8)	21 (7.9)	
Stairs/steps/escalator	59 (18.6)	15 (28.3)	44 (16.6)	
Wet Floor	49 (15.4)	3 (5.7)	46 (17.4)	
Ankle Twist	15 (4.7)	1 (1.9)	14 (5.3)	
Others	13 (4.1)	2 (3.8)	11 (4.2)	
**Time of fall**				
Morning	167 (52.5)	0 (0)	167 (63.0)	< 0.001*
Evening	95 (29.9)	44 (83.0)	51 (19.2)	
Night	56 (17.6)	9 (17.0)	47 (17.7)	
**Injuries/Injured body parts**				
Head	43 (14.4)	5 (9.8)	38 (15.3)	0.065
Face	54 (18.1)	9 (17.6)	45 (18.1)	
Neck	7 (2.3)	1 (2)	6 (2.4)	
Chest	17 (5.7)	1 (2)	16 (6.5)	
Abdomen	4 (1.3)	0 (0)	4 (1.6)	
Spine	11 (3.7)	3 (5.9)	8 (3.2)	
Upper Extremity	61 (20.4)	15 (29.4)	46 (18.5)	
Lower Extremity	96 (32.1)	19 (37.3)	77 (31.0)	
Foot	9 (3.0)	2 (3.9)	7 (2.8)	
None	39 (13.0)	5 (9.8)	34 (13.7)	
**Mode used for reaching hospital**				
Personal Car	196 (61.6)	49 (92.5)	147 (55.5)	< 0.001*
Ambulance	11 (34.9)	2 (3.8)	109 (41.1)	
Public Transport	7 (2.2)	2 (3.8)	5 (1.9)	
Careem/Taxi	4 (1.3)	0 (0)	4 (1.5)	

^*^Significant

The above table states the outcome of patients presented to ED due to the history of fall. At the end of one month, in the comorbid group, *n* = 20(7.5%) was expired but there was no mortality among people without any comorbid, whereas at the end of three months, there was an increase in mortality by 17% and 5.7% respectively (see Table 3).

**Table 3:** Outcomes of elderly patients with fall related injuries and risk of mortality (*n* = 318)

Characteristics	Total	Comorbidities *n* (%)		*p*-value
		**Without Comorbidity**	**With Comorbidity**	
	**318**	**53 (16.7%)**	**265 (83.3%)**	
**Discharge Status**				
Alive	298 (93.7)	53 (100)	245 (92.5)	0.039*
Expired	20 (6.3)	0 (0)	20 (7.5)	
**Outcome at three months**				
Alive	270 (84.9)	50 (94.3)	220 (83.0)	0.036*
Expired	48 (15.1)	3 (5.7)	45 (17.0)	

^*^Significant

Multivariable logistic regression shows that age, gender, assisting aid, history of previous fall, living alone, floor type, and reason of fall are significant predictors of mortality in elderly patients with fall related injuries. The risk of mortality among fall related male injured patients was 1.85 times (95% CI: 1.27–2.19) higher in comparison to females. Similarly, 1.48 times (95% CI: 1.20–2.10) higher in 80 years and above injured participants. The risk of mortality among fall related injuries elderly patients who wear eyeglasses was 1.57 times (95% CI: 1.17–2.23) higher and use walking aids was 1.60 times (95% CI: 1.19–2.37) greater compared to those who use hearing aids. Moreover, the risk of mortality amidst injured individuals, who had previous fall was 1.66 times (95% CI: 1.19–2.09) greater and those who lived alone had 1.19 times (95% CI: 1.04–1.78) more likely chance of falling than those who had no previous fall and were living with others. Furthermore, the risk of mortality among those who fell on concrete floor was 3.16 times (95% CI: 1.49–4.78) higher compared to those who fell on other surfaces. Similarly, the risk of mortality for those who fell due to blindness was 1.98 (95% CI: 1.48–2.70) compared to those who fell because of other reasons (see Table 4).

The article "Injuries and outcomes resulting due to falls in elderly patients presenting to the Emergency Department of a tertiary care hospital – a cohort study" was retracted in 2023. Reasons: errors in the text; plagiarized data; lack of ethics approval or compliance; no approval from a third party.

**Table 4:** Multivariable analysis of elderly participants with fall related injuries and risk of mortality

Characteristics	Crude Risk Ratio (95% CI)	Adjusted Risk Ratio (95% CI)
**Gender**		
Female	1	1
Male	2.60 (1.19–4.02)	1.85 (1.27–2.19)
**Age (Years)**		
< = 65 Years	1	1
66–80 Years	1.21 (1.11–1.85)	1.17 (1.08–1.77)
> 80 Years	2.70 (1.55–2.99)	1.48 (1.20–2.10)
**Employment Status**		
Unemployed	1	-
Employed	0.78 (0.30–1.47)	-
Own shop Rent	0.69 (0.24–1.39)	-
Housewife	0.39 (0.05–0.56)	-
Retired	0.77 (0.20–1.18)	-
**Education**		
Graduation	1	-
Illiterate	0.12 (0.01–0.52)	-
Primary	0.44 (0.23–0.97)	-
Secondary	1.02 (0.68–1.33)	-
Intermediate	1.85 (0.57–2.19)	-
Madrasa	0.25 (0.02–0.63)	-
**Assisting aid**		
Hearing aids	1	1
Eyeglasses	1.65 (1.47–2.14)	1.57 (1.17–2.23)
Walking aids	2.22 (1.92–4.62)	1.60 (1.19–2.37)
**Memory assessment**		
No	1	-
Yes	1.21 (0.88–1.65)	-
**Previous fall**		
No	1	1
Yes	2.44 (1.70–4.59)	1.66 (1.19–2.09)
**Living alone**		
No	1	1
Yes	1.14 (1.03–1.63)	1.19 (1.04–1.78)
**Place of fall**		
Road /outside home	1	-
Home	1.23 (0.41–1.69)	-
Bathroom	2.57 (1.27–4.23)	-
Stairs	2.06 (1.19–3.87)	-
Parking area	1.16 (0.50–1.90)	-
Prayer Place	1.13 (0.42–1.89)	-
Ground	2.39 (1.45–2.98)	-
Hospital	0.79 (0.37–1.59)	-
Other	1.34 (1.16–2.00)	-
**Floor type**		
Cement	1	1
Tile	3.02 (1.50–5.20)	2.57 (1.67–3.37)
Concrete	6.25 (2.95–15.57)	3.16 (1.49–4.78)
Carpets	1.68 (1.18–2.22)	1.60 (1.50–1.99)
Other	1.30 (1.07–1.72)	1.43 (1.22–1.85)
**Reason of fall**		
Stroke/ Seizures	1	1
Disbalance/Dizzy	2.66 (1.36–4.66)	1.46 (1.25–2.23)
Weakness	1.80 (1.22–2.56)	1.69 (1.40–2.61)
Visual (Blinded)	2.43 (2.00–5.30)	1.98 (1.48–2.70)
Wet Floor	1.84 (1.27–2.01)	1.57 (1.37–2.07)
Others	1.90 (1.48–2.29)	1.96 (1.49–2.28)
**Time of fall**		
Morning	1	-
Evening	0.88 (0.45–1.71)	-
Night	1.06 (0.97–1.96)	-
**Injuries/Injured body parts**		
Chest	1	-
Head & Neck	1.57 (0.97–3.37)	-
Face	1.96 (1.09–2.78)	-
Abdomen	1.06 (0.70–1.90)	-
Spine	1.33 (0.92–1.85)	-
Upper Extremity	2.39 (1.45–3.08)	-
Lower Extremity	0.99 (0.54–1.69)	-
Foot	1.04 (0.36–1.40)	-
**Mode used for reaching hospital**		
Personal Car	1	-
Ambulance	1.46 (0.45–3.23)	-
Public Transport	4.69 (1.70–6.26)	-
**Discharge status**		
Alive	1	-
Dead	2.39 (0.92–4.77)	-

The article "Injuries and outcomes resulting due to falls in elderly patients presenting to the Emergency Department of a tertiary care hospital – a cohort study" was retracted in 2023. Reasons: errors in the text; plagiarized data; lack of ethics approval or compliance; no approval from a third party.

## Discussion

Unintentional falls are a significant health problem for older people. The risk of an unintentional fall that results in mortality among the older population increases with age, thus demonstrating the need for intervention and awareness of this growing public health concern. Stevens et al. also showed that the risk for injury and mortality in older adults increases with age. There are intrinsic and extrinsic risk factors affecting a fall and its outcome. Considering the needs of the elderly, most of these factors are modifiable to prevent unfortunate events and their outcomes. We aimed to search primarily for the epidemiology and risk of mortality in older people with such fall-related injuries presenting to the Emergency Department [4, 17].

In this study, most of the patients were females, 55.1% of which had multiple comorbidities and fall-related injuries, comparable to the study conducted in Turkey by Tuba et al., which was around 70% [17]. A few other studies demonstrate that women are likely to sustain a fracture post fall resulting in compromised functionality. The falls were more prevalent among the female gender in comparison to males [11, 18]. This is likely due to the change in dynamics of female functionality as they are more active, which increases the likelihood of more frequent falls. On the other hand, a study published in the United States in 2015 favors that males have a higher risk of mortality after a fall [19]. Similarly, males had higher mortality than females (1.18 times higher in Austria, 2.4 higher in Slovakia) [19, 20].

In this study, falls were found to increase with age in patients with comorbidity, and almost 54% of individuals were between 60 to 80 years. Similar findings have been reported in a study conducted in US [21]. It was observed that most common were cardiovascular (93%), followed by endocrinological (79%), and cerebrovascular (51%). It was found in literature that elderly people with multiple comorbidities have higher chances of falling, which supports the findings of this study [22].

Most of the patients in this study (56%) were independent but were using assisting aids before fall, and their functionality was immensely affected post fall. It was also observed in this study that patients who had no comorbidities their activity of daily living assessed by (ADL/IADL) was better in comparison of people who had multiple comorbidities. A memory impairment assessment was done in this study and demonstrated that memory is in people with co-morbidities, and which is also observed to increase fall risk. Studies conducted in United States of America (USA) found that fall risk increases in elderly when there is dizziness, hearing impairment and vision loss [23, 24]. The previous history of falls was 31% especially among those with multiple comorbidities and elderly who found to be living alone 3.8% reported falls. This point is consistent and is significantly important because living alone posses a higher risk on elderly fall. Elliott et al., reported that there is a 50% higher chance of elderly to have a fall injury living alone compared to living with others [25].

The article "Injuries and outcomes resulting due to falls in elderly patients presenting to the Emergency Department of a tertiary care hospital – a cohort study" was retracted in 2023. Reasons: errors in the text; plagiarized data; lack of ethics approval or compliance; no approval from a third party.

The most frequent place of fall was the bedroom (40%) and bathroom (22%), staircase (5.7%) in elderly with comorbidities as reported in this study, the similar findings were reported in a study conducted in Thailand [26]. The various mechanisms of fall were found but the most common were disbalance (28.9%), weakness (14.5%), similar findings were found significant in Turkish study [27]. Gelbard et al. stated that most falls in elderly occur around the home, as elderly spend most of their time in their home, which was also reported in this study [4].

Moreover, in this study it was observed that after fall patients revisited almost 25% in ED and 63.58% revisited in the clinic at the end of first month. At the end of third month, 92.78% revisited altogether. McCusker et al. stated 19.3% revisited at the end of first month in ED [28]. The Friedmann et al. cohort study stated a revisit of 12% in the first 30 days and 19% in the third month [29]. As noticed previously, women suffer more falls, hence using more hospital services and more ED visits than males [11, 18]. Mortality resulting from falls in our study were associated with females, advanced age, and multiple comorbidities. Out of the three aforementioned factors, Sise et al. agree that fall related mortality increased 46% from 2002 to 2010 and was strongly associated with advanced age [30, 31].

In this study the death rate was higher in comparison to previous studies. A study conducted in the UK reported 7.9% compared to this study which reports 15% [29, 32]. It is also noted that patients with comorbidities suffered more deaths at one month 7.5% and at third month 17.5% though in international studies conducted in US it was 1.2% at one month and 15% at third month [5].

### Strength and limitations

This study is one of the few studies in Pakistan that reported factors and outcomes of fall injuries in elderly patients, and they are high risk population. This study has analyzed the association between comorbidities and fall among elderly which emphasizes on considering comorbidities when determining the prognosis of elderly patients presenting with falls This study is also the first to examine ED revisits and death of patients with fall related injuries. Moreover, a large sample size was used in the study. Despite strengths there are some limitations. This study was conducted in a private tertiary care hospital which has a standard of care, the results will be potentially different in public sector hospitals. Therefore, the results have limited generalizability.

The article "Injuries and outcomes resulting due to falls in elderly patients presenting to the Emergency Department of a tertiary care hospital – a cohort study" was retracted in 2023. Reasons: errors in the text; plagiarized data; lack of ethics approval or compliance; no approval from a third party.

## Conclusion

Elderly patients frequently revisit the ED and have high mortality rates sue to fall injuries. They are at high risk of morbidity and mortality due to falls. Efforts should be made to improve management of the underlying etiology of falls to prevent them in future. The factors that contribute to such incidences of fall should be identified, strategies and interventions should be planned to mitigate this risk. Further research needs to be done regarding managing the aetiology of elderly patients that suffered fall. There is also a need to review geriatric trauma care including the rehabilitation as well as acute management specially in LMICs like Pakistan. Moreover, the health care system in Pakistan needs to develop and provide post hospital health care services to the elderly patients after discharge.

## Data Availability

The data will be available at the reasonable request to the corresponding author at salman.soomar@aku.edu.

## Abbreviations

AKUH: Aga Khan University Hospital
CDC: Centre for Disease Control
ED: Emergency Department
UK: United Kingdom
USA: United States of America
WHO: World Health Organization
